The article "Effect of Moderate-Intensity Aerobic Exercise on Hepatic Fat Content and Visceral Lipids in Hepatic Patients with Diabesity: A Single-Blinded Randomised Controlled Trial" was retracted in 2023. Reasons: duplicated data; overlap with earlier publications; concerns about the data; concerns about the results or conclusions.

# Effect of Moderate-Intensity Aerobic Exercise on Hepatic Fat Content and Visceral Lipids in Hepatic Patients with Diabesity: A Single-Blinded Randomised Controlled Trial

**DOI:** 10.1155/2020/1923575

**Published:** 2020-04-11

**Authors:** Walid Kamal Abdelbasset, Shereen H. Elsayed, Gopal Nambi, Saud M. Alrawaili, Tamer E. Elnegamy, Mona A. Khalil, Sayed A. Tantawy, Gaber S. Soliman, Ahmed A. Ibrahim, Dalia M. Kamel

**Affiliations:** ^**1**^ Department of Physical Therapy and Health Rehabilitation, College of Applied Medical Sciences, Prince Sattam Bin Abdulaziz University, Alkharj, Saudi Arabia; ^2^Department of Physical Therapy, Kasr Al-Aini Hospital, Cairo University, Giza, Egypt; ^**3**^ Rehabilitation Sciences Department, Faculty of Health and Rehabilitation Sciences, Princess Nourah Bint Abdulrahman University, Riyadh, Saudi Arabia; ^**4**^ Department of Physical Therapy for Cardiovascular/Respiratory Disorders and Geriatrics, Faculty of Physical Therapy, Cairo University, Giza, Egypt; ^**5**^ Department of Biochemistry, Faculty of Medicine for Girls, Al-Azhar University, Cairo, Egypt; ^**6**^ Department of Physiotherapy, College of Medical and Health Sciences, Ahlia University, Manama, Bahrain; ^**7**^ Department of Physiotherapy, Centre of Radiation, Oncology and Nuclear Medicine, Cairo University, Giza, Egypt; ^**8**^ Department of Physical Therapy and Health Rehabilitation, College of Applied Medical Sciences in Al-Qurayyat, Jouf University, Sakakah, Saudi Arabia; ^**9**^ Department of Physical Therapy, College of Applied Medical Sciences, Hail University, Hail, Saudi Arabia; ^10^Department of Physiotherapy for Women's Health, Faculty of Physical Therapy, Cairo University, Giza, Egypt

## Abstract

**Objective:**

Limited studies have assessed the effect of moderate-intensity continuous aerobic exercise on hepatic fat content and visceral lipids in hepatic patients with diabesity. This study was designed to evaluate hepatic fat content and visceral lipids following moderate-intensity continuous aerobic exercise in hepatic patients with diabesity.

**Design:**

A single-blinded randomised controlled trial.

**Methods:**

Thirty-one diabetic obese patients with nonalcoholic fatty liver disease were recruited into this study. The patients were randomly classified into exercise and control groups, fifteen patients in the exercise group and sixteen patients in the control group. The exercise group received an 8-week moderate-intensity continuous aerobic exercise program with standard medical treatment, while the control group received standard medical treatment without any exercise program. Hepatic fat content and visceral lipids were assessed before and after intervention at the end of the study.

**Results:**

Baseline and clinical characteristics showed a nonsignificant difference between the two groups (*p* > 0.05). At the end of the intervention, the aerobic exercise showed significant improvements (serum triglycerides and low-density lipoproteins (LDLs), *p* ≤ 0.002, total cholesterol, *p*=0.004, visceral fats, *p*=0.016, glycated hemoglobin (HbA1C), *p*=0.022, high-density lipoproteins (HDLs), *p*=0.038, alanine transaminases (AL), *p*=0.044, intrahepatic triglyceride and HOMA-IR, *p*=0.046, and body mass index (BMI), *p*=0.047), while the control group showed a nonsignificant difference (*p* > 0.05). The postintervention analysis showed significant differences in favor of the aerobic exercise group (*p* < 0.05).

**Conclusions:**

Moderate-intensity continuous aerobic exercise reduces the hepatic fat content and visceral lipids in hepatic patients with diabesity. Recommendations should be prescribed for encouraging moderate-intensity aerobic exercise training, particularly hepatic patients with diabesity.

## 1. Introduction

Diabesity is a modern epidemic term used to depict the combination of type 2 diabetes mellitus (T2DM) and obesity. It is associated with different pathophysiological mechanisms such as insulin resistance and hyperinsulinemia [1]. Diabesity and fatty liver disease in combination with lower physical activity are potential causes to increase mortality and morbidity rates [2, 3]. Nearly a third of the world population experienced diabesity with dominant medical complications such as impairment of glucose, fat metabolism, and insulin sensitivity [4].

Accumulation of visceral adipose tissue and intrahepatic triglycerides (IHTG) is commonly one of the major characteristics of obesity that lead to impairments of cardiovascular function, metabolism, and insulin sensitivity [5, 6]. Ordinarily, the reduction of IHTG is subsequently related to an increase in metabolism and restore normal blood glucose in T2DM [7]. Few documents approved the positive influences of exercise training and dietary control on IHTG with no definitive medical prescription reducing hepatic fat [8].

Nonalcoholic fatty liver disease (NAFLD) is associated with serum hypertriglyceridemia and impairment of liver lipoprotein metabolism [9]. Exercise training and dietary control reduce IHTG and improve metabolic function in patients with NAFLD [10, 11]. Poor documents explained the role of exercise training in the treatment of NAFLD. Previous studies found a nonsignificant correlation between the level of physical activity and the changes in hepatic histology in those patients. However, these studies observed the high measure of maximal oxygen uptake (VO_2peak_) in mild NAFLD, confirming the vital function of exercise training in the management of this type of patients [12]. Also, other studies provided that physical exercise and dietary control reduce steatosis [13–15], liver fat content [16–18], depression status [19, 20], ventilatory marker dysfunctions [21], and slow down progression of T2DM [22].

Restricted studies assessed the clinical effects of moderate-intensity continuous aerobic exercise in hepatic patients with diabesity. Our study hypothesized that moderate-intensity continuous aerobic exercise could reduce hepatic fat content and visceral lipids in hepatic patients with diabesity. Therefore, this study was designed to assess the hepatic fat content and visceral lipids following moderate-intensity continuous aerobic exercise in those patients.

## 2. Subjects and Methods

### 2.1. Subjects

Thirty-one NAFLD patients with diabesity were included in this single-blinded randomised controlled trial between August and December 2017. All study patients were referred by the physician for endemic disease in accordance with the department's approval to the outpatient physical therapy clinic, Cairo University Hospitals. Patients were included in the study if they were clinically diagnosed with T2DM, Obesity class II-III (BMI ≥ 35 kg/m^2^), and NAFLD. They have followed in the endemic diseases, endocrine, and diabetes outpatient clinics and received their medications such as metformin, omega-3 fatty acids, and pentoxifylline. NAFLD has been diagnosed on the basis of the Asia-Pacific region guidelines for the diagnosis of NAFLD [23]. Patients were randomly divided into exercise and control groups. The exercise group received moderate-intensity continuous aerobic exercise with standard medical treatment, while the control group received standard medical treatment without exercise intervention. The patients were excluded if they have a severe life-limiting illness, cardiac disorders, neuromuscular dysfunctions, orthopedic, and endocrinal complications that could disturb exercise programs. This study was approved on 03/06/2017 by the scientific review committee of the Physical Therapy Department, Cairo University Hospitals (No.: PT/2017/00-019). All patients signed informed consent before starting the study program.

### 2.2. Sample Size Estimation

To nullify a type II error, a preliminary power analysis (power, 0.80; *α* = 0.05; effect size, 0.5) was performed. The sample size was estimated according to the IHTG value. Early studies provided that aerobic exercise training exhibited a significant mean difference of the IHTG value 1.76 with a standard deviation of 2.2 [24]. In accordance with that study, 13 patients were required in each group. 32 patients in the exercise and control groups were included into account for the dropout rate of 20%.

### 2.3. Randomisation

Of the 37 patients, 32 individuals were worthy of enrolling in the study. 3 individuals were not eligible by the criteria of the study and 2 individuals withdrew from the study without reasons. Randomization was performed before participating in the study of the evaluator utilizing secured envelopes, which included a piece of colored sheet regarding the aerobic exercise group and a piece of white sheet regarding the control group. The flow diagram exhibiting the patients who participated in the study is demonstrated in Figure 1.

## 3. Procedure of the Study

### 3.1. Evaluation

Each patient was assessed for IHTG, visceral lipids, lipid profile, insulin sensitivity, glycated hemoglobin (HbA1c), and alanine transaminases (AL) before and after intervention by the same evaluator who was blinded to the study group allocation and the aim of the study. The procedure and the nature of the study were explained for all patients before intervention.

### 3.2. Radioimaging Evaluation

Magnetic resonance imaging (MRI, 3T scanner, General electric, WI) was used to assess hepatic fat by chemical shift imaging. All patients were evaluated using the body coil in the supine position. During imaging, each patient was recommended to take one hold breath and three separated images of slice couples were obtained for the hepatic cell. The proportionate of IHTG to water was calculated using the equation of 100 × (triglyceride signal amplitude)/(water signal amplitude). This study used MRI as it is identified, validated, and designed as the commonest precise noninvasive method investigating the level of fatty liver in subjects with T2DM [25].

### 3.3. Biochemistry Evaluation

After fasting 10 hrs, blood samples were obtained in the early morning and analyzed biochemically to assess total cholesterol, total triglycerides (TGs), low-density lipoproteins (LDLs), high-density lipoproteins (HDLs), AL, and HbA1c.

### 3.4. Intervention

Exercise and control groups were recommended for home-based exercises such as walking and stretching exercise. Also, both groups were informed to adhere to the recommendations of their physicians during the study program.

### 3.5. Exercise Protocol

Each patient in the exercise group was recruited to a moderate-intensity continuous aerobic exercise program 3 times weekly for 8 weeks, the duration of the exercise was nearly 40–50 minutes. All patients were informed to prevent eating 2 hours before the exercise program to nullify exercise-related respiratory dysfunction. The moderate-intensity continuous exercise program consisted of 5-minute warming-up followed by a cycling Ergometer (MonarkRC6, Novo Langley, USA) with continuous intensity at 60–70% of the maximum heart rate (max HR) and the exercise program ended with 5-minute cooling-down.

### 3.6. Data Analysis

The statistical Package for Social Science v.22 (SPSS, Chicago, IL, USA) was used for data analysis. Descriptive analysis was summarized using means and standard deviations for normally distributed data. Normality was checked using the Kolmogorov–Smirnov test. Inferential statistics assessed differences of the study measures including (IHTG, visceral lipids, plasma lipids, and HbA1c) using student's *t* test; independent *t* test between the two study groups and paired *t* test were conducted to calculate the differences within each group. Values of *p* < 0.05 were considered statistically significant.

## 4. Results

Of the 32 patients who enrolled in the study program, one patient was excluded from the statistical analysis because of irregular attendance in the exercise program. Thirty-one NAFLD patients with diabesity (17 men and 14 women) were analyzed; their age was ranged 45–60 years. The exercise group included 15 patients (8 men and 7 women), while the control group included 16 patients (9 men and 7 women). Baseline and clinical characteristics exhibited nonsignificant differences between the exercise and control groups before the study intervention (*p* > 0.05) as described in Table 1.

Comparing between before and after 8 weeks intervention, mean values showed significant improvement in the exercise program (triglycerides and LDL, *p* ≤ 0.002; total cholesterol, *p*=0.004; visceral fats, *p*=0.016; HbA1C, *p*=0.022; HDL, *p*=0.038; AL, *p*=0.044; intrahepatic triglyceride and HOMA-IR, *p*=0.046; and BMI, *p*=0.047), while they showed nonsignificant differences in the control group (*p* > 0.05) as detailed in Table 2. The pre- and post-percentage changes were (IHTG = 18.6%, HOMA-IR = 17.02%, TGs = 9.61%, AL = 8.29%, LDLs = 7.21%, total cholesterol = 6.62%, BMI = 6.5%, visceral fats = 6.27%, HbA1c = 6.25%, and HDLs = 6.13%) in the exercise group versus (IHTG = 0.89%, HOMA-IR = 3.75%, TGs = 1.11%, AL = 4.36%, LDLs = 0.21%, total cholesterol = 1.38%, BMI = 0.83%, visceral fats = 1.44%, HbA1c = 2.98%, and HDLs = 3.37%) in the control group as described in Figure 2.

Comparing the mean values between the exercise and control groups after 8 weeks of follow-up, there was a significant difference in favor of the exercise group (*p* < 0.05) as described in Table 2.

## 5. Discussion

The findings of the study endorsed that moderate-intensity continuous aerobic exercise training reduces the body mass index, hepatic fat content, visceral lipids, and HbA1c in hepatic patients with diabesity particularly NAFLD. The results of the present trial emphasized that moderate-intensity continuous exercise three times per week for eight weeks (cycling exercise at 60–70% of max HR for 40–50 minutes) exhibited a definite decrease of hepatic triglycerides, visceral adipose fat, and body mass index. Similar results were reported in the prior articles of exercise training on NAFLD patients [16–18, 26, 27].

The reduction of hepatic triglycerides with moderate-intensity aerobic exercise is mechanically related to the decrease of circulating lipids and insulin resistance. This study emphasizes the importance of moderate-intensity aerobic exercise in populations with excess hepatic lipids. Despite the fact that the extreme visceral adipose fat has come from the circulating fatty acids and secretions of adipocytokines, which increase insulin resistance and intrahepatic lipids [28], the precise physiological relation between liver metabolism and visceral lipids remains obscure. Obviously, the continuity of controlled metabolism in the present trial is an alarming assumed hepatic lipid reduction and the forceful link between hepatic insulin resistance and intrahepatic lipids [29]. Evidence approved that the reduction of IHTG is importantly required to lower insulin resistance and blood glucose levels [29, 30].

In consent to the present study findings, Aoi et al. provided that 20-minute submaximal heart rate cycling or running exercise aspired to 20-minute warm-up/cool-down three sessions per week for 4 weeks results in a reduction in insulin resistance and blood glucose levels in patients with T2DM [31].

Various researches evaluated the ideal exercise intensity to improve basic and comprehensive metabolic panels. O'Donovan et al. investigated the influences of moderate-intensity exercise (cycling exercise at 60% VO_2max_ three times per week for 24 weeks) and high-intensity exercise (cycling exercise at 80% VO_2max_ three times per week at 24 weeks) on blood glucose levels and insulin sensitivity. Aerobic exercise at an intensity of 60% and 80% VO_2max_ was sufficient to increase insulin sensitivity and decrease plasma glucose levels [32].

Also, Benatti et al. explained that 60-minute treadmill aerobic exercise daily for twelve weeks at 70% VO_2max_ (80% max HR) leads to a significant reduction in body weight, insulin resistance, visceral lipids, and abdominal obesity [33]. In addition, this study approved that aerobic exercise without reduction of body weight also reduced visceral and abdominal fat.

Moreover, prior studies verified that 50–60 minutes of daily aerobic exercise for 4 weeks (beginning with 60–65% max HR and ending by 80–85% max HR) resulted in improvement of insulin sensitivity, glucose oxidation, and visceral lipids [34]. Similarly, Abdelbasset et al. approved that cycling exercise with 80% to 85% VO_2max_ and interval at 50% VO_2max_ for 40 minutes 3 times weekly for eight weeks showed a fluent decrease of hepatic triglycerides, visceral fats, and insulin resistance in diabetic obese patients with NAFLD [35, 36].

Regardless of ALT increase is the usual prediction of hepatic dysfunction [37], changes in plasma ALT are not a predictor of hepatic histological changes [38]. Also, our study found a remarkable decrease in plasma ALT in the exercise group and approved a beneficial clinical practice of moderate-intensity continuous exercise in NAFLD patients with diabesity.

This randomised controlled trial has some strengths. It establishes strong evidence for accenting the important role of moderate aerobic exercise in diabetic obese patients with NAFLD. Also, it clarifies that moderate-intensity continuous aerobic exercise (40–50 minutes, three times per week at 60–70% of max HR), reduces hepatic fat content, visceral lipids, plasma ALT, and plasma glucose levels and improves insulin sensitivity in NAFLD patients with diabesity. Appropriate control of the fatty liver disease has to commence with exercise adherence, consequently, as moderate-intensity aerobic exercise modulates insulin sensitivity by an improvement of free fatty acid metabolism in exercised skeletal muscles. Hence, free fatty acid oxidation and insulin sensitivity result in the increase of glucose-lipid metabolism. Also, regular exercise training results in the expressive decrease in hepatic fat content by the increase in energy expenditure and skeletal fat oxidation and decrease in visceral lipids.

The present study has some limitations. Firstly, the lack of intermediate and long-term assessment. Secondly, home-based exercise and dietary intake were not supervised. Further researches have to include a large sample size to evaluate different exercise intensities on diabetic obese patients with NAFLD.

## 6. Conclusions

Moderate-intensity continuous aerobic exercise reduces hepatic fat content and visceral lipids in hepatic patients with diabesity. Extra connotations for clinical applications have to be dedicated to adhere to the moderate-intensity continuous aerobic exercise program among hepatic patients, particularly fatty liver patients with diabesity.

## Figures and Tables

**Figure 1:** Flow diagram of the study.

**Figure 2:** Pre- and post-percentage changes in exercise and control groups.

**Table 1:** Baseline and clinical characteristics of the two groups before intervention.

Parameters	Exercise group (*n* = 15)	Control group (*n* = 16)	*p* value
Age (years)	54.9 ± 4.7	55.2 ± 4.3	0.854
Sex, *n* (%)			
Men	8 (53.3)	9 (56.2)	0.843
Women	7 (46.7)	7 (43.8)	
BMI (kg/m^2^)	36.7 ± 3.4	35.9 ± 5.3	0.629
Clinical characteristics			
Intrahepatic triglyceride (%)	12.9 ± 4.2	11.2 ± 5.1	0.349
Visceral adipose fat (cm^2^)	181.7 ± 13.5	179.8 ± 14.4	0.708
Total triglycerides (mg/dL)	196.5 ± 12.6	198.1 ± 11.8	0.718
Total cholesterol (mg/dL)	193.2 ± 8.8	188.3 ± 8.4	0.123
HDL-cholesterol (mg/dL)	37.5 ± 3.4	38.5 ± 3.3	0.421
LDL-cholesterol (mg/dL)	98.4 ± 5.7	95.2 ± 4.8	0.101
AL (IU/L)	44.6 ± 5.1	43.5 ± 4.6	0.533
HOMA-IR	4.7 ± 1.4	4.8 ± 1.5	0.704
HbA1c (%)	6.4 ± 0.5	6.7 ± 0.6	0.143

Sig.: significance level at *p* < 0.05. BMI: body mass index. HDL: high-density lipoproteins. LDL: low-density lipoprotein. AL: alanine transaminase. HOMA-IR: homeostatic model assessment-insulin resistance. HbA1c: glycated hemoglobin.

**Table 2:** Outcome measures before and after intervention in the exercise and control groups.

Parameters	Exercise group (*n* = 15)			Control group (*n* = 16)		
	Before	After	*pvalue*	Before	After	*p* value
BMI (kg/m^2^)	36.7 ± 3.5	34.3 ± 2.8	0.047	35.9 ± 5.3	36.2 ± 5.5^*∗*^	0.827
Intrahepatic triglyceride (%)	12.9 ± 4.2	10.5 ± 1.5	0.046	11.2 ± 5.1	11.1 ± 5.2^*∗*^	0.899
Visceral adipose fat (cm^2^)	181.7 ± 13.5	170.3 ± 10.6	0.016	179.8 ± 14.4	177.2 ± 12.8^*∗*^	0.455
Total triglycerides (mg/dL)	196.5 ± 12.6	177.4 ± 9.7	<0.001	198.1 ± 11.8	200.3 ± 11.6	0.462
Total cholesterol (mg/dL)	193.2 ± 8.8	180.4 ± 8.7	0.004	188.3 ± 8.4	185.7 ± 8.1^*∗*^	0.219
HDL-cholesterol (mg/dL)	37.5 ± 3.4	39.8 ± 2.3	0.038	38.5 ± 3.3	37.2 ± 4.1^*∗*^	0.174
LDL-cholesterol (mg/dL)	98.4 ± 5.7	91.3 ± 4.6	0.002	95.2 ± 4.8	95 ± 4.6^*∗*^	0.867
AL (IU/L)	44.6 ± 5.1	40.9 ± 4.5	0.044	43.5 ± 4.6	45.4 ± 4.7^*∗*^	0.113
HOMA-IR	4.7 ± 1.4	3.9 ± 0.5	0.046	4.8 ± 1.5	4.98 ± 1.8^*∗*^	0.671
HbA1c (%)	6.4 ± 0.5	6.0 ± 0.4	0.022	6.7 ± 0.6	6.5 ± 0.5^*∗*^	0.312

Sig. : significance level at *p* < 0.05. ^*∗*^; significant differences between the two groups after intervention. BMI: body mass index. HDL: high density lipoproteins. LDL: low density lipoprotein. AL: alanine transaminase. HOMA-IR: homeostatic model assessment-insulin resistance. HbA1c: glycated hemoglobin.

## Data Availability

This study is a single-blinded randomised controlled trial, the data involved are available from the corresponding author upon request, and privacy-related parts of the patient will not be provided.
